# Value of Combining Optical Coherence Tomography with Fundus Photography in Screening Retinopathy in Patients with High Myopia

**DOI:** 10.1155/2022/6556867

**Published:** 2022-04-11

**Authors:** Yingjuan Hao, Shiyang Liu, Zhimin Yu

**Affiliations:** ^1^Department of Ophthalmology, Nanjing Tongren Hospital, School of Medicine, Southeast University, Nanjing 211102, Jiangsu Province, China; ^2^Department of Ophthalmology, Central Hospital Affiliated to Shandong First Medical University, Jinan, 250013, Shandong Province, China

## Abstract

**Objective:**

To explore the value of combining optical coherence tomography (OCT) with fundus photography in screening retinopathy in patients with high myopia.

**Methods:**

By means of retrospective study, 40 high myopia patients with retinopathy treated in our hospital from January 2020 to January 2021 were selected as the study group, and 40 healthy individuals in the same period were included in the control group. All patients received traditional ophthalmic examination, and accepted fundus fluorescence imaging, OCT, and fundus photography examination step by step by the same operator. After that, three physicians read the slides by the double blind method, and took the results of fundus fluorescence imaging as the gold standard to analyze the diagnostic efficacy of OCT, fundus photography and their combination.

**Results:**

The clinical data and examination results showed that no statistical differences in general data including patients' mean age, gender ratio, and educational degree between the study group and the control group were observed (*P* > 0.05), and the nerve thickness above/below the optic disk and temporal/nasal nerve thickness of the optic disk of the study group were significantly different from those of the control group (*P* < 0.001); the sensitivity, specificity, positive predictive value (PPV), negative predictive value (NPV), and accuracy rate of diagnosis of combining OCT with fundus photography were respectively 95.0%, 97.5%, 97.4%, 95.1%, and 96.3%, which were significantly higher than OCT or fundus photography alone (*P* < 0.05); and for combined examination, AUC (95%CI) = 0.963 (0.000–1.000).

**Conclusion:**

Combining OCT with fundus photography can effectively identify high myopia patients with retinopathy, which is conducive to improving clinical positive ratio and providing objective basis for treatment.

## 1. Introduction

High myopia is defined as ametropia with over 600 degrees of myopia. The disease is characterized by extension of optic axis, usually accompanied by various degrees of fundus pathology, including posterior scleral staphyloma, leopard shaped fundus, and macular hemorrhages, which may lead to blindness in severe cases [1, 2]. According to a survey by the World Health Organization in 2018, China has 600 million myopic patients, nearly 10.0% of students are highly myopic, with the proportion increasing with age, and the incidence of high myopia in high school students can reach 17.6% [3, 4]. Relevant data predict that the myopia rate in the Chinese population over 5 years of age will increase to 66.0% over the next two decades, while the incidence of high myopia may climb to 10.0%–13.0% [5, 6]. Because high myopia seriously threatens the sustainable development of China's economic society, it is extremely important to strengthen research on the means of screening. Currently, clinical diagnosis of high myopia related ophthalmic diseases is generally performed by direct ophthalmofundoscope, preset lens, and fundus fluorescence imaging [7, 8]. Such imaging modality is recognized as the gold standard for the examination of high myopia, which can clearly outline the vessel morphology, elevate the vessel contrast, and clarify the morphological characteristics and axial length of fundus retina in patients with high myopia, thereby providing valuable basis for clinical diagnosis. However, it cannot measure retinal thickness or clearly exhibit the lesion structure and layers, indicating certain limitations. With the continuous optimization of imaging technology, precise measurement of retinal thickness in high myopia patients in vitro has been achieved, such as optical coherence tomography (OCT), which can be used to acquire high-resolution cross-sectional images and clearly present the tomographic structure of each tissue in the eye with the near-infrared diffuse optical tomography, while repeatedly measuring the thickness of different layers of the retina [9]. In addition to OCT, fundus photography also has the advantages of noninvasion, convenience, and repeatability and is characterized by economic applicability, presenting potential for broad promotion at the basic level. In particular, the introduction of nonmydriatic fundus photography technology has provided more possibilities for patients who are not suitable for mydriasis. Scholars Pawar Bhargavi and others showed that nonmydriatic fundus photography screening for diabetic retinopathy had a Youden index of 79.1 and Kappa of 80.7 [10], indicating that fundus photography is valuable in retinal examination to some extent. Combining OCT with fundus photography may be conducive to further improving the positive ratio of retinopathy in high myopia patients and providing objective basis for early treatment. Based on this, the study explored the diagnostic efficacy of the combination, with the results reported as follows.

## 2. Materials and Methods

### 2.1. Study Design

It was a retrospective study conducted in our hospital from January 2020 to January 2021 to explore the value of combining OCT with fundus photography in screening retinopathy in high myopia patients. It was a double-blind study, meaning that neither the research objects nor researchers understood the trial grouping, and the study designer was responsible for arranging and controlling the full trial.

### 2.2. Enrollment of Study Objects

Inclusion criteria: (1) patients met the diagnosis criteria for high myopia [11], with diopter > -6.0D, length of optic axis ≥26.0 mm, and intraocular pressure between 10.0 and 21.0 mmHg; (2) patients met the diagnosis criteria for retinopathy; (3) patients were treated in our hospital in the whole course and had complete clinical data; and (4) patients were at least 18 years old.

Exclusion criteria: (1) patients could not go along with ophthalmic examination; (2) patients quit the study before completion; (3) patients had other severe organic diseases, or other diseases that might affect the study results; (4) patients had history of eye injury; (5) patients had history of refractive surgery, internal eye surgery, or retinal laser treatment; (6) patients had refractive stromal opacity that affected examination; and (7) patients were not suitable for fundus fluorescence imaging, OCT or fundus photography.

### 2.3. Inclusion of Study Objects

According to the inclusion and exclusion criteria, 40 high myopia patients with retinopathy treated in our hospital from January 2020 to January 2021 were selected as the study group, and 40 healthy individuals in the same period were included in the control group. The study only conducted to one affected eye of each patient. After collecting and analyzing the general data of the study objects, it was found that no statistical differences in general data including mean age, gender ratio, and educational degree between the study group and the control group were observed (*P* > 0.05), meaning that they could be enrolled as the study objects.

### 2.4. Moral Consideration

The study met the principles in the *World Medical Association Declaration of Helsinki (2013)* [12]. After enrollment, the study team explained the study purpose, meaning, contents and confidentiality to the patients and asked the patients to sign the informed consent.

### 2.5. Criteria for Quitting the Study

For those who had one of the following situations and were judged by the study team as not suitable to continuously accept the study, their case records would be retained but would not be used for data analysis. (1) Those with severe disease progression during the trial and (2) those who were unwilling to proceed with the clinical trial and proposed the requirement of quitting the clinical trial to the study team.

## 3. Methods

All patients received the traditional ophthalmic examination, to be specific, the visual acuity was examined by the international logarithmic visual acuity chart, the length of optic axis was measured by ophthalmology ultrasound diagnosis instrument made by Tomey Corporation (NMPA Registration (I) no. 20203160149), the optometry and calculation of diopter and best corrected visual acuity (BCVA) were performed by auto-refractomer made by Carl Zeiss Meditec AG (NMPA Registration (I) no. 20152162139), and the intraocular pressure was measured by noncontact tonometer made by Carl Zeiss Meditec AG (NMPA Registration (I) no. 20192160241), and by means of double blind, three physicians read the slides of the examinations. If one of the diagnostic results from OCT or fundus photography was positive, it was considered as definite diagnosis; if the results from both examinations were negative, it was considered diagnosis undetermined.

### 3.1. Fundus Fluorescence Imaging

Instrument: Fundus camera CLARUS made by Carl Zeiss Meditec, Inc. (NMPA Registration (I) no. 20202160524).

Steps for inspection: patients were inquired about their history of drug allergy, liver and kidney function, and blood pressure, and those with normal blood pressure should have imaging indications. Patients' pupils should be fully dilated before imaging, then 10 ml of 0.1% fluorescein sodium was administered by slow intravenous injection to forearm elbow vein (Shandong Bausch&Lomb Freda Pharmaceutical Co. Ltd.; NMPA approval no. H20093096), during which the patients were closely monitored for allergic reactions, if no allergic reactions 5 min later, 3 ml of 20% fluorescein sodium was quickly administered via intravenous injection, and 10 s after injection, optic papilla, retinal vessels, macular region, and peripheral retina and choroid were under multidirectional observation for imaging changes for 8–15 min.

#### 3.1.1. OCT

Instrument: Tomey Cornea/Anterior Segment CASIA2 (NMPA Registration (I) no. 20203160473).

Steps for inspection: Patients' pupils should be fully dilated before examination, internal eye fixation was suitable for patients with visual acuity ≥0.5 or central fixation, and external eye fixation was suitable for patients with visual acuity <0.5 or noncentral fixation. OCT instrument was applied for horizontal or vertical linear scan, and for convention test, the scan was performed through foveal centralis with four lines, 6.0 mm in length, 45° interval, and 2.0 mm in depth. The scan direction was adjusted according to the lesion situation, and the scan quality was ensured to be above 30 dB each time.

#### 3.1.2. Fundus Photography Examination

Instrument: Fundus camera CLARUS made by Carl Zeiss Meditec, Inc. (NMPA Registration (I) no. 20202160524).

Steps for inspection: patients were adapted to the dark environment for 5 min, then fundus photography was performed to take two 45° fundus photographs centered on the macula and optic disc of the affected eye.

### 3.2. Observation Criteria

1. General data: study objects' gender, age, height, body mass, BMI, educational degree, and the affected eye for study, mean diopter, and BCVA of patients in the study group.
2. Diagnostic results from different diagnosis methods: the diagnostic results from OCT, fundus photography, and their combination were recorded.
3. Diagnostic efficacy of different diagnosis methods: ① sensitivity: number of true positive cases/(number of true positive cases + number of false negative cases) *∗* 100%; ② specificity: number of true negative cases/(number true negative cases + number of false positive cases) *∗* 100%; ③ positive predictive value (PPV): number of true positive cases/(number of true positive cases + number of false positive cases); and ④ negative predictive value (NPV): number of true negative cases/(number of false negative cases + number of true negative cases).
4. ROC curve: ROC curves of different diagnosis methods were plotted by SPSS20.0, and AUC (95%CI) was recorded.

### 3.3. Statistical Processing

In this study, the data processing software was SPSS20.0, the picture drawing software was GraphPad Prism 7 (GraphPad Software, San Diego, USA), the items included were enumeration data and measurement data, the methods used were X^2^ test and *t*-test, and differences were considered statistically significant at *P* < 0.05.

## 4. Results

### 4.1. Patients' General Data

The clinical data and examination results showed that no statistical differences in general data including patients' mean age, gender ratio, and educational degree between the study group and the control group were observed (*P* > 0.05), and the nerve thickness above/below the optic disk and temporal/nasal nerve thickness of the optic disk of the study group were significantly different from those of the control group (*P* < 0.001). See Table 1.

### 4.2. Diagnostic Results from Different Diagnostic Methods

For diagnostic results from different diagnosis methods, seeTables 2–4.

### 4.3. Diagnostic Efficacy of Different Diagnosis Methods

The sensitivity, specificity, PPV, NPV, and accuracy rate of diagnosis of combining OCT with fundus photography were respectively 95.0%, 97.5%, 97.4%, 95.1%, and 96.3%, which were significantly higher than OCT or fundus photography alone (*P* < 0.05). See Table 5.

### 4.4. ROC Curves of Different Diagnosis Methods

For OCT, fundus photography, and their combination respectively, AUC (95%CI) = 0.837 (0.744–0.931), 0.725 (0.611–0.839), and 0.963 (0.000–1.000). See Figure 1.

## 5. Discussion

High myopia refers to ametropia characterized by extension of optic axis and retinal and choroidal degeneration in the fundus, and high myopia patients present with various degrees of structural and functional retinal changes and thinning of the retinal thickness, with thinning and degeneration of retina in the posterior pole being more pronounced [13, 14]. Previous studies considered high myopia to be associated with increased diopter but often ignored retinopathy conditions, resulting in patients losing optimal treatment timing. Recent reports have shown that the influence of retinal thickness is not limited to mechanical traction caused by the extension of the optic axis, and fundus lesions in the posterior pole can also lead to abnormal choroidal vascular perfusion, which can affect the outer retinal blood supply and metabolism, and finally cause the reduction of the number of nucleated cell layers, the gradual atrophy of the retina and choroid, and irreversible reduction of central vision [10, 15, 16]. Therefore, active screening for high myopic retinopathy with imaging techniques and providing patients with corresponding treatment on this basis may effectively reduce the risk of irreversible visual function damage.

Because highly myopic patients have a higher diopter accompanied by astigmatism, vitreous opacity and other features, and their fundus lesions are not easily visible under direct test lens, so fundus fluorography is the best method for screening fundus lesions in them [17, 18]. Fundus fluorescence imaging can present retinal and choroidal blood circulation, and dynamically and objectively record small changes in the center and periphery of the macula in affected eyes of patients with high myopia, which is beneficial for providing an objective basis for clinical treatment. However, fundus fluorescence imaging is an invasive examination with complicated operation steps and high risk coefficient, and the research by Sugihara Kazunobu found that such examination had low acceptance [19], which cannot meet the potential screening needs in China with a large population base and high incidence of myopia. Compared with fundus fluorescence imaging, the novel OCT technique has the advantages such as noninvasion and easy operation, which can quantitatively analyze the retinal structure through noncontact ways, so that physicians can observe the retinal tomographic imaging horizontally, vertically, and via radiation, and obtain more precise retinal information, thereby providing more basis for evaluating retinopathy [20–22]. The study found that the nerve thickness above/below the optic disk and temporal/nasal nerve thickness of the optic disk of the study group were statistically different from those of the control group (*P* < 0.001), demonstrating that OCT could effectively monitor the retina thickness changes in the posterior pole, thus offering new ideas for determining the progression of pathological myopia.

Scholars Dhami Abhinav and others found that the noncontact nature of OCT makes it more acceptable to patients, especially in minor patients, and patient satisfaction with OCT is significantly higher than that of routine examination [23]. However, the sensitivity of OCT alone in detecting high myopia retinopathy is only 80.0%, presenting certain improvement potential. In view of the large myopic patient population in China, techniques combined with OCT should equally have the possibility of large generalizability at the basic level, so fundus photography was jointly adopted in this study. Previously fundus photography was usually performed by 7-field stereography after mydriasis, which was tedious and time-consuming [11]. With the constant upgrade of related technology, mydriasis free fundus photography has been applied in clinic, which presents easy operation and ideal patient compliance. The study results showed that the sensitivity, specificity, PPV, NPV, and accuracy rate of diagnosis of combining OCT with fundus photography were respectively 95.0%, 97.5%, 97.4%, 95.1%, and 96.3%, which were significantly higher than OCT or fundus photography alone (*P* < 0.05). And the ROC curves further demonstrated that for combined examination, AUC (95%CI) = 0.963 (0.000–1.000), showing that the combination had good diagnostic efficacy and could meet the application demands in the Chinese market.

To sum up, combining OCT with fundus photography can effectively identify high myopia patients with retinopathy, which is conducive to improving the clinical positive rate and has a better promotion value than that of fundus fluorescence imaging, thus meeting the demand of screening retinopathy in patients with high myopia in China.

## Figures and Tables

**Figure 1:** ROC curves of different diagnosis methods.

**Table 1:** Comparison of patients' general data.

Group	Study group	Control group	X^2^/*t*	*P*
Gender				
Male	22	22	0.000	1.000
Female	18	18		
Mean age	36.30 ± 17.80	36.58 ± 15.56	0.075	0.941
Mean height (cm)	174.65 ± 12.65	174.70 ± 12.78	0.018	0.986
Mean body mass (kg)	62.32 ± 2.65	61.98 ± 2.47	0.594	0.555
BMI (kg/m^2^)	21.66 ± 1.23	21.70 ± 1.25	0.144	0.886
Educational degree				
Primary school and below	10	12	0.251	0.617
Senior high school	18	20	0.201	0.654
Junior college and above	12	8	01.067	0.302
Affected eye			−	-
Left eye	25	-		
Right eye	15	-		
Mean diopter (D)	−11.23±−1.23	-	-	-
BCVA	0.81 ± 0.07	-	-	-
Nerve thickness above optic disk (*μ*m)	115.65 ± 5.23	147.65 ± 8.98	19.475	<0.001
Nerve thickness below optic disk (*μ*m)	117.65 ± 5.65	138.65 ± 7.55	14.084	<0.001
Optic disk temporal nerve thickness (*μ*m)	68.45 ± 4.65	88.40 ± 6.50	15.788	<0.001
Optic disk nasal nerve thickness (*μ*m)	54.98 ± 4.55	73.98 ± 7.55	13.632	<0.001

**Table 2:** Diagnostic results from fundus photography.

Fundus photography	Fundus fluorescence imaging		
	Positive	Negative	Total
Positive	30	12	42
Negative	10	28	38
Total	40	40	80

**Table 3:** Diagnostic results from OCT.

OCT	Fundus fluorescence imaging		
	Positive	Negative	Total
Positive	32	6	38
Negative	8	34	42
Total	40	40	80

**Table 4:** Diagnostic results from combination of OCT and fundus photography.

OCT combined with fundus photography	Fundus fluorescence imaging		
	Positive	Negative	Total
Positive	38	1	39
Negative	2	39	41
Total	40	40	80

**Table 5:** Diagnostic efficacy of different diagnosis methods.

Group	Sensitivity (%)	Specificity (%)	PPV (%)	NPV (%)	Rate of accuracy (%)
OCT	80.0 (32/40)	85.0 (34/40)	84.2 (32/38)	81.0 (34/42)	82.5 (66/80)
Fundus photography	75.0 (30/40)	70.0 (28/40)	71.4 (30/42)	73.7 (28/38)	72.5 (58/80)
OCT combined with fundus photography	95.0 (38/40)	97.5 (39/40)	97.4 (38/39)	95.1 (39/41)	96.3 (77/80)

## Data Availability

Data to support the findings of this study are available on reasonable request from the corresponding author.
